# Antihypertensive and Vasorelaxant Effects of *Citrus aurantifolia* Linn. Fruit: Proposed Mechanisms

This article has been retracted.

**DOI:** 10.1155/2022/5871424

**Published:** 2022-05-20

**Authors:** Syed Nasir Abbas Bukhari, Alamgeer, Sumera Saeed, Mulazim Hussain Asim, Hafiz Muhammad Irfan, Hasan Ejaz, Mervat A. Elsherif, Kashaf Junaid

**Affiliations:** ^1^Department of Pharmaceutical Chemistry, College of Pharmacy, Jouf University, Sakaka, Al Jouf 72388, Saudi Arabia; ^2^Punjab University College of Pharmacy, University of the Punjab, 54000 Lahore, Pakistan; ^3^College of Pharmacy, University of Sargodha, 40100 Sargodha, Pakistan; ^4^Department of Clinical Laboratory Sciences, College of Applied Medical Sciences, Sakaka, Jouf University, Al Jouf 72388, Saudi Arabia; ^5^Chemistry Department, College of Science, Jouf University, Al Jouf 72388, Sakaka, Saudi Arabia

## Abstract

**Background:**

*Citrus aurantifolia* Linn. fruit, a natural dietary item, has long been used traditionally to treat hypertension in Pakistan. The current research work aims to explore the effect on blood pressure and its mechanisms.

**Methods:**

The aqueous methanol extract of plant fruit was used to evaluate hypotensive/antihypertensive, vasorelaxation, and safety profiles. Moreover, the *in vitro* inhibitory effect of AMECA on phosphodiesterase was also evaluated.

**Results:**

In hypotensive studies, extracts of *Citrus aurantifolia* fruit exhibited a concentration-dependent reduction in SBP, DBP, MAP, and heart rate. A similar effect has been observed on anesthetized rats, but the effects exerted by the extract were not altered significantly in the presence of L-NAME, atropine, captopril, and propranolol. Moreover, in coronary arteries, the extract significantly potentiated relaxations induced by cGMP- and cAMP-dependent relaxing agonists. When exposed to PDEs, the extract concentration dependently subdued cGMP-hydrolyzing activity of different PDEs with IC50 values of 40–130 *μ*g/mL.

**Conclusion:**

It is conceivable that extracts obtained from *Citrus aurantifolia* fruit produced hypotensive and antihypertensive effects in rats. The extract elicited endothelium-independent vasorelaxation, possibly by acting directly on smooth muscles of the coronary artery and by increasing cGMP and cAMP via nonselective inhibition of vascular PDEs.

## 1. Introduction

Hypertension, a leading cause of cardiovascular diseases, is famous as the “silent killer” due to its asymptomatic nature [1]. It is one of the major contributors of the global disease burden [2]. A number of researchers reported that hypertension as a leading cause of death affects every cultural society all around the world [3]. Contemporary medicines effectively reduced the mortality of cardiovascular diseases. However, the long-term use of these medicines is beyond the reach of the common population, especially in 3rd-world countries. Synthetic medicines are one of the good sources of drugs in modern medicine, are expensive, and have several side effects [4]. Therefore, different options of the treatment are need of the time [5]. Natural products have played a vital role in drug development for cancer, infectious diseases, multiple sclerosis, and cardiovascular diseases [6–9]. A lot of plants are reported to have a significant effect on blood pressure [10–13].

Pakistan has a rich inheritance of medicinal plants that are being extensively used for curing various diseases by local people. *Citrus aurantifolia* Linn. (Rutaceae), an indigenous plant in Pakistan, has been used traditionally to treat hypertension, cough, headache, and sore throat and also as an antiseptic, anthelmintic, antiarthritic, tonic, astringent, diuretic, and appetite stimulant [14–18]. The fruit and other parts of the plant are being used in Ayurveda, Siddha, and many other folk systems for the cure of different ailments. It has been used for the treatment of hypertension by the people in Enderta, Northern Ethiopia, and Edo State, Nigeria [19, 20]. Pharmacologically, this plant has been investigated for its antibacterial, antimicrobial, antioxidant, anticancer, and anthelmintic activities [21, 22]. The fruit contains vitamin C, minerals, flavonoids, and other important phytochemicals. The purpose of the current study was to evaluate the antihypertensive effect of *Citrus aurantifolia* fruit extract in normotensive and hypertensive rats. It was further aimed to evaluate its potential to affect vascular tone and underlying mechanisms of vasorelaxation.

## 2. Materials and Methods

### 2.1. Chemicals

Atrial natriuretic peptide, bradykinin, forskolin, glucose, isoproterenol, methanol, sodium nitroprusside, U46619, atropine, captopril, propranolol, and L-NAME were obtained from Sigma. All the other chemicals used in this study were of analytical grade and purchased from different commercial sources.

### 2.2. Experimental Animals

Sprague-Dawley rats (200–250 g) and albino BALB/c mice (28–35 g) of either sex were kept in the animal house of the University of Sargodha, Sargodha, Pakistan, in a controlled environment with a humidity of 65–70% at a 12 h light and dark cycle. The animals were delivered a standard diet and water *ad libitum*. For vascular reactivity studies, fresh porcine hearts were obtained from an abattoir. Animals were provided with all standard nutritional and housing conditions according to principles for laboratory animal use and care, and it was assured that there should be minimum animal suffering during the study.

### 2.3. Ethical Approval

The animal handling and study protocols were approved by the Institutional Animal Ethical Committee, College of Pharmacy, University of Sargodha, Pakistan (No. IAEC/UOS/2015/23). During the experimental work, it was assured that the test animal suffered minimal pain or discomfort.

### 2.4. Plant Material and Preparation of the Extract

*Citrus aurantifolia* fruits were obtained from the herbal market in Sargodha, Pakistan, and identified by Assistant Professor Dr. Amin-Ullah (Department of Botany, University of Sargodha). For further research reference, an herbarium specimen (# A-8047) was submitted to the herbarium, Department of Botany, University of Sargodha. An aqueous methanol (30:70) extract of fruit juice was generated using the cold maceration method. The fruit juice (10 L) was soaked in an aqueous methanol mixture (10 L) at room temperature for 72 h with random shaking and then filtered and evaporated using a rotary evaporator. The aqueous methanol extract of *Citrus aurantifolia* (AMECA) was air-dried to get a honey-brown semisolid mass soluble in distilled water. The extract was preserved in an airtight container at 4°C [5, 23].

### 2.5. Study in Normotensive Rats

#### 2.5.1. Evaluation of Acute Hypotensive Effect of *Citrus aurantifolia* Linn

Rats were assigned to different groups. Groups I, II, and III received 0.25, 0.5, and 0.75 g/kg of the oral *Citrus aurantifolia* aqueous methanol extract, respectively. The heart rate and basal blood pressure were recorded at predetermined time points after extract administration with the help of noninvasive blood pressure (NIBP) equipment (IN125, AD Instruments, Australia). For testing, the rat was put in an NIBP restrainer and the sensor cuff was fixed on the tail. The tail cuff was adjusted to 200 mmHg systolic blood pressure, released slowly, and recorded with the PowerLab data acquisition system. The SBP, MAP, and HR were measured via pulse tracing, whereas the diastolic blood pressure was evaluated from SBP and MAP using the following equation [5, 24, 25]:

(1) $$\begin{array}{c} \text{DBP}=\frac{3\text{MAP}-\text{SBP}}{2}. \end{array}$$

#### 2.5.2. Screening Hypotensive Effect in Anesthetized Normotensive Rats

Rats were anesthetized with 70–90 mg/kg of sodium thiopental intraperitoneally. The trachea was exposed by gently removing the steroid muscle to facilitate respiration. A polyethylene catheter attached with a pressure transducer was inserted into the left common carotid artery, while the right jugular vein was cannulated for intravenous administration of drugs [26]. After stabilization, various doses of the extract (5, 10, 15, 20, 25, and 30 mg/kg) were injected with a time gap of at least 10 min between each dose. The effects of the extract on various parameters of blood pressure (SBP, DBP, MAP, and HR) were studied using the PowerLab data acquisition system [27].

#### 2.5.3. Investigation of the Possible Hypotensive Mechanism in Anesthetized Normotensive Rats

To explore the underlying mechanisms of hypotension, a selected dose of the extract (20 mg/kg) was given for 40 min in anesthetized rats previously treated with atropine at a dose of 2 mg/kg, propranolol at a dose of 1 mg/kg, captopril at a dose of 2.5 mg/kg, and L-NAME at a dose of 20 mg/kg for 10 min before the injection of the extract [28]. The effect on SBP, DBP, MAP, and HR was recorded through the PowerLab data acquisition system [29, 30].

### 2.6. Study in Hypertensive Rats

#### 2.6.1. Effect of *Citrus aurantifoli*a Linn. in Glucose-Induced Hypertensive Rats

Rats were divided into 2 groups randomly. Group I was fed with glucose contrary to tap water for 3 consecutive weeks, while group II received glucose and AMECA at 0.75 g/kg dose for the same time. Throughout the study period, all animals were given a standard diet. The heart rate and blood pressure were determined at predetermined time points of 0, 1, 2, and 3 weeks with a noninvasive blood pressure-measuring apparatus by the tail-cuff method as described earlier [5, 25].

#### 2.6.2. Vascular Reactivity Studies

Vasorelaxation is one of the key mechanisms of antihypertensive drugs. Several drugs produce antihypertensive effects via their action on blood vessels. The aim of this experiment was to explore whether this exact same procedure produces a hypotensive/antihypertensive effect via relaxation of vessels. For this purpose, fresh pork hearts were obtained to isolate coronary artery. The porcine coronary arteries were cleaned of connective tissues, cut into rings of 4-5 mm in length, and suspended in organ baths containing saturated 95% O_2_ and 5% CO_2_ Krebs bicarbonate solution at 37°C. The composition of Krebs bicarbonate in mmol/L is MgSO_4_ 1.18, KCl 4.7, NaCl 119, NaHCO_3_ 25, KH_2_PO_4_ 1.18, D-glucose 11, and CaCl_2_ 1.25 at pH 7.4. The rings were contracted twice with 80 mmol/L KCl after an equilibration period of 90 min. Rings were then contracted with 1–60 nmol/L of thromboxane mimetic U46619 followed by an endothelium integrity checkup with 0.3 *μ*mol/L bradykinin. The rings were again contracted with U46619 after 30 min of washout. The concentration response curve was developed by the cumulative addition of 0.0001–0.1 mg/mL aqueous methanolic extract of *Citrus aurantifolia* fruit in both intact coronary artery rings and denuded endothelium [31].

#### 2.6.3. Study on the Role of ANP, SNP, FC, and Isoproterenol in Vascular Reactivity of the Tested Extract

For evaluation of these effects, endothelium-denuded coronary artery rings were placed in Kreb's bicarbonate solution. Before contractions with U46619 coronary artery rings were incubated with 0.01mg/mL of tested extract, and ANP, SNP, FC, and isoproterenol were added cumulatively (1 nM-1*μ*M). Similarly, the same concentration-response curves were designed with the same test samples without extract, and the percentage relaxations produced by these test samples were measured [31].

#### 2.6.4. Determination of PDE Inhibitory Effects of the Tested Extract

The experiment was performed as described by previously published studies. In brief, the bovine aorta was used to isolate PDE isoforms. PDE1 was evaluated in the presence of cGMP in basal and calmodulin-activated states. The PDE3 and PDE4 were evaluated in the presence of rolipram and an excess of cGMP, respectively, so that during chromatographic separation, cross-contamination should be avoided. At last, PDE5 activity was determined with cGMP (1 *μ*M) using EGTA (1 mM). IC50 values of extracts at various concentrations were recorded via regression analysis [31, 32].

### 2.7. Acute Toxicity Testing

Both male and female albino mice were randomly distributed into 5 groups (*n* = 2). Group I received 10 mL/kg of normal saline serving as control, while groups II, III, IV, and V were fed with an ascending order of extract doses (1, 1.5, 2, and 2.5 g/kg, respectively). After administration of the extract, animals were continuously observed for mortality for 24 h. If no mortality was observed, then another five groups of the animals were selected and were treated again with different doses of the tested extract in the increasing order (3, 3.5, 4, 4.5, and 5 g/kg) intraperitoneally. The maximum dose did not kill any mouse, and the minimum dose that killed any mouse was noted and LD_50_ was recorded [33].

### 2.8. Statistical Analysis

The data are expressed as mean ± SEM using GraphPad software. The comparison of different values was made using Student's *t*-test, and two-way ANOVA has been applied with Bonferroni's posttest. *p* < 0.05 < 0.01 was taken as statistically significant.

## 3. Results

### 3.1. Acute Hypotensive Effect in Normotensive Rats

The extract dose of 0.25 g/kg reduced DBP and MAP after 2 and 4 h as compared to the control (0 h). However, this dose did not significantly alter the heart rate. Moreover, 0.5 g/kg of the extract abridged SBP after 2 h, while DBP and MAP were reduced after 2 and 4 h of its administration. Also, this dose brought a reduction (*p* < 0.01) in heart rate within 2 h of its administration and 0.75 g/kg produced a significant (*p* < 0.001) fall in heart rate and blood pressure after 2 and 4 h after administration in comparison to control, as shown in Table 1.

### 3.2. Effect in Hypertensive Rats

The effect of the aqueous methanol extract of *Citrus aurantifolia* in glucose-treated hypertensive rats is illustrated in Table 2. The extract at 0.75 g/kg dose produced a significant drop in SPB, DPB, MAP, and HR of treated rats in comparison to control from the 1^st^ to 3^rd^ week of treatment in all three models.

### 3.3. Investigation of Possible Hypotensive Effects in the Anesthetized Rat

Administration of various doses (5, 10, 15, 20, 25, 30 mg/kg) of AMECA in anesthetized normotensive rats showed a dose-dependent significant hypotensive effect as shown in Figure 1.

### 3.4. Investigation of Possible Hypotensive Mechanisms in Anesthetized Rats

Pretreatment of L-NAME and atropine did not change the hypotensive effect of AMECA. Similarly, the administration of propranolol and captopril also did not affect the hypotensive response produced by AMECA as expressed in Figure 2.

### 3.5. Effects of the Extract on Porcine Coronary Artery Rings

The aqueous methanol extract of *Citrus aurantifolia* fruit (0.0001–0.3 mg/mL) showed a concentration-dependent relaxant effect on intact and denuded endothelium coronary artery rings as reflected in Figure 3. The EC_50_ values of 0.0439 mg/mL and 0.0416 mg/mL were found for the intact endothelium and denuded endothelium, respectively. The elimination of the endothelium had no influence on the relaxation of artery rings. At all test doses, a nonsignificant change in relaxation was produced by the extract in the intact endothelium and denuded rings.

### 3.6. *Citrus aurantifolia* Extract Potentiated Coronary Artery Relaxations by cGMP- and cAMP-Elevating Agents

0.01 mg/mL of the extract significantly produced concentration-dependent response curves of 0.1 nM to 0.1 *μ*M in the trial natriuretic peptide ANP and 1 nM to 0.3 *μ*M in sodium nitroprusside (SNP). The maximum relaxation produced by ANP was 38%, while in the presence of extracts, 60% relaxation was achieved (Figures 4(a) and 4(b)).

0.01 mg/mL dose of the extract significantly altered the concentration-dependent response curve with 1 nM-1 *μ*M concentration of forskolin and isoproterenol as compared to control. The change in EC_50_ for the extract for forskolin was 0.397–0.152 *μ*M, while this change for isoproterenol was 0.142–0.076 *μ*M, as depicted in Figures 4(c) and 4(d).

### 3.7. *Citrus aurantifolia* Extract Showed an Inhibitory Effect on Vascular Phosphodiesterase (PDE)

The methanol extract of *Citrus aurantifolia* fruit nonselectively inhibited the vascular isoforms of PDE such as PDE5 with an IC_50_ value of 48.59 ± 1.4 *μ*g/mL, PDE4 with an IC_50_ value of 64.78 ± 1.4 *μ*g/mL, PDE3 with an IC_50_ value of 105.46 ± 1.5 *μ*g/mL, and PDE1 with an IC_50_ value of 104.60 ± 1.2 *μ*g/mL in its basal states and PDE1 calmodulin with an IC_50_ value of 80.14 ± 1.2 in the activated state, as depicted in Figure 5.

### 3.8. Acute Toxicity Testing of the Extract

The lethal dose (LD_50_) of the extract was calculated at 3.0 g in mice, and before death, the animals exhibited signs of convulsion as well.

## 4. Discussion

The present study shows that the aqueous methanol extract of *Citrus aurantifolia* (AMECA) produces acute and chronic hypotensive effects in normotensive rats. A similar pattern was shown by the extract when tested in anesthetized normotensive rats using an invasive blood pressure-measuring technique. The extract prevented the rise in DBP, SBP, MAP, and heart rate in glucose-fed hypertensive rats.

The antihypertensive effect of the tested extract was more pronounced than its effect on normotensive rats, which supports previous findings that hypertensive rats show an exaggerated response to depressor stimuli compared to normotensive rats [34]. During mechanistic studies in normotensive rats, the results of the current study suggested that the hypotensive effect of AMECA is not linked with inhibition of angiotensin-converting enzyme or activation of muscarinic receptors. Furthermore, in light of the present findings, it could also be proposed that the adrenergic system or nitric oxide synthesis is also not a mechanism of the possible hypotensive effect of AMECA. Previous findings revealed that glucose administration causes a rise in blood pressure in experimental rats through multiple mechanisms such as sodium retention, dyslipidemia, fluid volume expansion, and increase in sympathetic overactivity [35]. The present study demonstrated that the tested extract significantly reduced the rise in glucose-induced blood pressure. Our findings are in accordance with previously published studies [29].

The prolonged use of glucose produces free radicals and reactive oxygen species, which are the main motives for high blood pressure [35, 36]. Antioxidants are famous for reducing reactive oxygen species. The juice of *Citrus aurantifolia* has been reported to be rich in ascorbic acid and flavonoids. Furthermore, it displayed antioxidant activity [37, 38]. In the present study, the tested drug might have reduced glucose-induced hypertension because of its antioxidant activity by reducing reactive oxygen species. In the glucose-hypertensive model, it might be due to the decrease in oxidative stress. It has been reported that ascorbic acid reverses oxidative damage and vascular dysfunction [39]. Therefore, the preventive effect of AMECA on increasing blood pressure may be due to these antioxidants which have the ability to counteract the harmful effects of free radicals.

It has been reported that vascular muscle plays a significant part in vasorelaxation and various drugs produce an antihypertensive effect by instigating the relaxation of blood vessels. Therefore, *Citrus aurantifolia* fruit extract was further investigated to appraise its potential to modify the vascular tone. It is proved that endothelium regulates vascular tone through relaxant and contractile factors [40]. The findings of the present study revealed that vasorelaxation effect of the tested extract is possibly mediated via its direct effect on vascular smooth muscles. It was noted that the relaxation response was produced in intact and endothelium-denuded coronary arteries and there was no significant difference between them, indicating the endothelium-independent effects.

Since U46619 has been described to perform through thromboxane-prostanoid receptors, the tested extract might have produced a relaxation effect by interacting with the attachment ability of U46619 with T/P receptors. Moreover, the vascular tone has been controlled by the cyclic nucleotide amount in smooth muscles; therefore, *Citrus aurantifolia* fruit extract was also studied on relaxations induced by cGMP or cAMP. The endothelium-independent vasodilators like atrial natriuretic peptide and sodium nitroprusside, isoproterenol, and forskolin cause vasorelaxation by activating the cGMP and c-AMP-dependent relaxing pathways, respectively, in smooth muscles [41]. As a potent vasorelaxant, the atrial natriuretic peptide is activated by guanylyl cyclase while SNP prompts relaxation of smooth muscles, and these pathways lead to increased cGMP levels [42]. This cGMP-mediated relaxation may also be due to a reduction in intracellular Ca^2+^ amount via sarcoplasmic reticulum activation, Na^+^/K^+^ ATPase, Ca^2+^ ATPase, and different potassium channels [43–46]. Moreover, a decline in the contractile apparatus sensitivity to Ca^2+^ has been described as a cGMP-mediated relaxation mechanism [47]. Isoproterenol is well known to produce relaxation through the cAMP pathway activation, whereas forskolin directly stimulates adenyl cyclase to produce vasodilatation effect [48]. Another reason is that this effect can be because of protein kinase-A (PKA) activation that phosphorylates various proteins involved in different special effects, for instance, the rise of Ca^2+^ uptake into the sarcoplasmic reticulum and inhibition of myosin light chain kinase activation of Ca^2+^ efflux [49, 50].

In the current study, it was found that the *Citrus aurantifolia* fruit extract significantly shifted the concentration-dependent response curve of these endothelium-independent vasodilators to the left. The data obtained have indicated that the *Citrus aurantifolia* fruit extract has potentiated relaxations indicating their stimulating effect on the formation of cGMP and cAMP.

It has been previously reported that PDE inhibitors enhance the relaxant effects of forskolin, isoproterenol, and SNP [51]. In the present study, the tested extract also potentiated the relaxations induced by these vasodilators. These results indicate that the hypotensive effect of the extract might have also been attributed due to its inhibitory effect on PDEs.

Therefore, the extract was further investigated to evaluate its direct inhibitory effect using purified vascular smooth muscles having 4 major types of PDEs: PDE1 generally hydrolyzes cGMP and PDE3 hydrolyzes cAMP and can also hydrolyze cAMP, while PDE4 and PDE5 specially hydrolyze cAMP and cGMP, respectively [52]. In the current study, the extract significantly inhibited all types of PDEs. These findings provide direct evidence that the tested extract has the potential to inhibit vascular PDEs and has an effect on various PDE isozymes, leading to endothelium-independent vasorelaxation through the accumulation of cAMP and cGMP levels. These findings are consistent with the previous studies [53]. In acute toxicity testing, the methanolic extract (3 g) was found safe.

## 5. Conclusion

It is conceivable from the study that *Citrus aurantifolia* may exert its hypotensive/antihypertensive effects through multiple mechanisms in rats. According to the present findings, the major mechanism of the antihypertensive effect could be its vasorelaxation effect. The extract produced vasorelaxation through endothelium-independent mechanisms via increasing both cGMP and cAMP levels through inhibition of vascular PDEs. However, further studies are necessary to explore the exact mechanism of the antihypertensive effect including further vasorelaxation mechanisms. A detailed phytochemical study of the tested extract is also required to find the exact secondary metabolite which is responsible for antihypertensive, vasorelaxation, and PDE inhibitory effects.

## Figures and Tables

**Figure 1:** Effect of the aqueous-methanol extract of *Citrus aurantifolia* on SBP, DBP, MAP, and HR. (a) Effect of AMECA on blood pressure. (b) Effect of different doses of AMECA on the heart rate of anesthetized rats. Values are presented as mean ± SEM. Here, SBP denotes the systolic blood pressure, DBP denotes the diastolic blood pressure, and MAP denotes the mean arterial pressure. Two-way ANOVA has been applied with Bonferroni's posttest using GraphPad Prism version 6.0 and ^*∗∗∗*^*p* < 0.001, compared to control.

**Figure 2:** Effect of the *Citrus aurantifolia* aqueous methanol extract on the mean arterial pressure of anesthetized rats. The animals in the control group were treated with normal saline (0.1 mL/kg), and all other groups received an aqueous methanol extract of *Citrus aurantifolia* (CA) at 20 mg/kg. They were previously treated with atropine at a dose of 2 mg/kg, propranolol at a dose of 1 mg/kg, captopril at a dose of 2.5 mg/kg, and L-NAME at a dose of 20 mg/kg for 10 min before injection of the extract.

**Figure 3:** *Citrus aurantifolia* fruit causes relaxation in porcine coronary artery rings. E−: denuded endothelium and E+: intact endothelium.

**Figure 4:** Effects of the aqueous methanol extract of *Citrus aurantifolia* fruit (0.01 mg/mL) on relaxation produced by (a) atrial natriuretic peptide, (b) sodium nitroprusside, (c) forskolin, and (d) isoproterenol in U46619 precontracted denuded porcine coronary artery rings. ^*∗*^*p* < 0.05, ^*∗∗*^*p* < 0.01, and ^*∗∗∗*^*p* < 0.001 in comparison to control.

**Figure 5:** Inhibitory effects of different amounts of the extract on vascular PDE isoforms.

**Table 1:** Acute hypotensive effect of the aqueous methanol extract of *Citrus aurantifolia* fruit.

Parameters	0.25 g/kg	0.50 g/kg	0.75 g/kg
SBP (mmHg)			
0 h	124.13 ± 0.44	123.88 ± 0.55	123.63 ± 0.56
2 h	120.25 ± 0.59	113.63 ± 1.59^*∗*^	95.75 ± 1.61^*∗∗*^
4 h	123.75 ± 0.49	118.00 ± 1.49	103.8 ± 3.20^*∗∗*^
6 h	123.38 ± 0.53	122.63 ± 0.38	122.75 ± 0.49

DBP (mmHg)			
0 h	92.68 ± 0.48	92.62 ± 0.39	93.54 ± 0.32
2 h	67.45 ± 3.79^*∗∗*^	67.69 ± 3.04^*∗∗*^	62.81 ± 1.61^*∗∗*^
4 h	79.13 ± 3.29^*∗*^	72.13 ± 1.95^*∗∗*^	74.25 ± 2.11^*∗∗*^
6 h	93.56 ± 0.23	93.96 ± 0.24	94.57 ± 0.30

MAP (mmHg)			
0 h	103.16 ± 0.25	103.04 ± 0.25	103.56 ± 0.18
2 h	85.69 ± 2.72^*∗∗*^	79.75 ± 1.75^*∗∗*^	76.38 ± 0.89^*∗∗*^
4 h	94.00 ± 2.28^*∗*^	87.00 ± 1.16^*∗∗*^	84.13 ± 1.13^*∗∗*^
6 h	103.50 ± 0.16	103.58 ± 0.14	103.96 ± 0.22

HR (beats/min)			
0 h	382.10 ± 0.50	382.66 ± 0.31	382.6 ± 0.45
2 h	381.75 ± 1.13	375.88 ± 1.44	368.3 ± 1.89^*∗*^
4 h	383.50 ± 1.18	374.50 ± 0.91^*∗*^	373.6 ± 0.98^*∗*^
6 h	382.06 ± 0.71	383.58 ± 0.14	381.3 ± 0.67

Values are presented in mean ± SEM. ^*∗*^*p* < 0.01 and ^*∗∗*^*p* < 0.001 in comparison to control (0 h).

**Table 2:** *Citrus aurantifolia* extract significantly reduced blood pressure in hypertensive rats.

Parameters	Glucose	
	Control	Treated
SBP (mmHg)		
Week 0	124.7 ± 1.5	122.5 ± 0.6
Week 1	146.7 ± 2.5	116.7 ± 1.1^*∗*^
Week 2	161.1 ± 2.6	110.2 ± 1.9^*∗*^
Week 3	177.7 ± 1.7	87.6 ± 2.6^*∗*^

DBP (mmHg)		
Week 0	92.9 ± 0.9	101.5 ± 2.2
Week 1	122.5 ± 1.9	97.4 ± 1.3^*∗*^
Week 2	127.9 ± 5.2	84.9 ± 2.1^*∗*^
Week 3	133.3 ± 1.9	64.5 ± 1.9^*∗*^

MBP (mmHg)		
Week 0	103.6 ± 0.3	108. ± 1.6
Week 1	130.6 ± 0.9	130.9 ± 0.7^*∗*^
Week 2	139.0 ± 2.8	93.4 ± 1.2^*∗*^
Week 3	148.1 ± 1.3	72.2 ± 0.6^*∗*^

HR (beats/min)		
Week 0	383.6 ± 0.3	382.9 ± 0.7
Week 1	394.4 ± 1.1	371.4 ± 1.3^*∗*^
Week 2	420.3 ± 3.1	357.1 ± 1.1^*∗*^
Week 3	433.1 ± 3.0	342.2 ± 3.2^*∗*^

Values are presented as mean ± SEM. ^*∗*^*p* < 0.01 in comparison to control.

## Data Availability

The data used to support the findings of this study are included within the article.
